# Quality of Services Based on Intelligent IoT WLAN MAC Protocol Dynamic Real-Time Applications in Smart Cities

**DOI:** 10.1155/2021/2287531

**Published:** 2021-10-31

**Authors:** Abbas Alnazir, Rania A. Mokhtar, Hesham Alhumyani, Elmustafa Sayed Ali, Rashid A. Saeed, S. Abdel-khalek

**Affiliations:** ^1^Department of Electrical Engineering, College of Engineering, Red Sea University, Port Sudan, Sudan; ^2^Department of Computer Engineering, College of Computers and Information Technology, Taif University, P.O. Box 11099, Taif 21944, Saudi Arabia; ^3^Department of Electronics Engineering, College of Engineering, Sudan University of Science and Technology, Khartoum 1111, Sudan; ^4^Department of Mathematics, College of Science, Taif University, P.O. Box 11099, Taif 21944, Saudi Arabia

## Abstract

The future directions and challenges for 6G-enabled wireless communication for IoT applications are mainly focused on quality of service (QoS). The selection criteria of mobility management (MM) protocol are mainly the total duration of the delay and packet loss rate during the MM procedure. This is called intelligent handover (IH) to designate a relay with a minimum delay. To solve the problem of handover, media access control (MAC) protocols are used to provide an intelligent protocol for QoS in real-time application in mobility. Moreover, changing the parameter to find the best protocol for mobile stations in WLAN is a good choice. This paper proposed a new QoS structure for the point coordination function that is based on a new intelligent enhanced distribution coordination function that suites with dynamic real-time applications and services. The paper addresses the distributed coordination function (DCF) with QoS-based intelligent mobility management in stations and other scenarios with enhanced distribution coordination function (EDCF) to find the result of throughput, retransmission attempts, delay, and data droop. In this paper, the remote topology comprises a few remote stations and one base station within the remote LAN. All remote stations are found that each station can distinguish a transmission from any other station, and there is portability within the proposed intelligent framework.

## 1. Introduction

Wireless LAN technology is the most successive edge network for different communication applications, which can provide simple and flexible network connectivity, in addition to the efficient ability of system scalability and deployment. Recently, IoT WLAN had attention to be more deployed to provide many services and be a part of smart city infrastructure to enable multimedia in real-time service applications. The future directions and challenges for 6G-enabled wireless communication for IoT applications are mainly focusing on the quality of services (QoS). In WLAN applications, quality of service (QoS) is considered an important issue in evaluating the performance of real-time services. The technology known as IEEE802.11 MAC provides a suitable mechanism to control the channel access in WLAN [1–3]. The IoT WLAN MAC is depending on two mechanisms, a coordination distributed function (DCF), and an optional point coordination function (PCF). DCF enables distribution of the channel access according to the carrier sense access with collision avoidance (CSMA/CA). PCF is based on the polling approach to provide control channel access.

The concept of MAC protocol is related to the potential improvement in QoS, which relates to several characteristics that must be taken into consideration such as packet loss, delay, bandwidth, and data traffic over the network [4]. WLAN provides a data transmission system to enable accessing between independent network and user devices wirelessly. Generally, WLAN is used to provide a communication link between the wired backbone networks to a group of wireless devices, which have independent resources and services. Another concept is micromobility that describes the movement of a mobile node between two attachment points on the same network [5]. Due to device mobility, handover management is required to perform stable communications based on the device locations and WLAN access points. For that, some functions must necessarily have a protocol authorizing the mobility management, citing the transfer of packets, the update of ways or roads, the management of handovers, the support of inactive mobiles, the management of addresses, authentication and security mechanisms, and so on [6–9].

When considering IoT WLAN networks, it was found that the quality of service varies from one application to another, depending on the bandwidth used and the factors related to delay and loss of data. The standard IEEE 802.11 MAC cannot be able to provide an efficient QoS performance in multimedia applications. This is because multimedia requires that MAC serve all transmission frames with the same priority level [10]. Therefore, new technology has been identified with the ability to deal with applications that require high QoS and are known as IEEE 802.11e. An enhanced distributed function (DCF) mechanism is used for IEEE 802.11e to provide QoS prioritization for WLAN applications [11]. This paper proposed a new QoS structure for the point coordination function that is based on a new intelligent enhanced distribution coordination function that suites with dynamic real-time applications and services, for example, smart city-based internet-of-thing (IoT) services, that is, RT surveillances, unmanned transportations and vehicles, smart management system for energy, and city control and monitoring rooms for environmental and security.

The remainder of this paper is organized as follows: Section 2 is discussed on intelligent IoT WLAN MAC QoS-related work and problematic issues.  Section 3 discusses the proposed theoretical model of enhanced distribution coordination function (EDCF).  Section 4 is discussed the system-level simulation results and discussions. Finally, the paper is concluded, and the future directions and challenges for 6G-enabled wireless communication with dynamic QoS were given.

## 2. Related Works and Motivation

Tall information rates at the physical layer at versatility have ended up conceivable in remote communication [12]. MAC strategy is considered an improvement for single-channel remote systems in WLAN, which enables the sharing of common radio channels. It provides an effective utilization of the accessible transmission capacity and ensures the fulfillment of QoS prerequisites of both information and real-time applications in portability [13]. Services related to real-time applications, such as those related to video and audio communications, need WLAN with a higher quality of service and better performance.

In [10], it reviewed the concept of IEEE 802.11 as a working group to supplement IEEE 802.11e WLAN, which provides better quality of service (QoS) to multimedia and other real-time applications. The authors also analyzed the IEEE 802.11e and IEEE 802.11 WLAN Intelligent MAC protocols and compare them in terms of QoS performance, latency, throughput, and packet loss. The comparison results show that IEEE 802.11e has outperformed the QoS of IEEE 802.11 in channel allocation and management conditions [14]. However, IEEE 802.11 protocol is found better than IEEE 802.11e in collision resolution when the network is highly congested.

In [15], it proposed a Markov model to analyze the EDCF performance for IEEE802.11e. The author provides the present extensive performance evaluation for EDCF in terms of throughput and access delay related to the flows in RTS/CTS mode [16]. Moreover, the study presents the quantitative analysis for the parameters of arbitration interframe space, and contention window (CW), in addition to their effect on QoS.

In [17], the authors proposed and evaluated the enhanced distributed coordination function (EDCF) and compare it with 802.11 original standards. From the evaluation, the authors reviewed that EDCF enables to access channel frames with different priorities. The study also presents the concept of contention-free burst (CFB) [18] and its ability to enable multiple frame transmissions during a single transmission opportunity. The evaluation results show that EDCFS enables different traffic to be provided by differentiated channel access. Moreover, the use of CFB helps improve the performance of EDCF and ensures high WLAN network throughput with acceptable delays. In [19], the authors proposed reviewing the main properties of distribution coordination function (DCF) and point coordination function (PCF) in IEEE802.11 IOT WLAN MAC and showed that the two mechanisms can support better QoS [20].

According to the importance of EDCF for different WLAN based on IEEE802.11 [21], we consider that the EDCF mechanism in IEEE 802.11e enables it to enhance the WLAN QoS, especially for shared wireless media applications. The paper aims to evaluate the performance of EDCF and EDCF protocols in mobility [22]. The paper will study the elementary perceptions and problems of wireless networks that can enhance WLAN quality of service (QoS) and examine various existing Intelligent IoT WLAN MAC protocols of WLAN. In addition, the study will implement and compare efficient mechanisms that can improve the QoS of WLAN. In our study, various parameters will be evaluated for EDCF protocols such as network load, data dropped, and access delay [23].

## 3. Intelligent IoT WLAN MAC Layer

MAC protocol is used to enhance the operation of channel media accessing, which is considered as a logical entity that enables to control and coordinate the system and device access to the radio channels [24]. The MAC performs the operations related to frames to handle data traffic between the PHY layer and the wired network.  Figure 1 shows the frame of packet format accessed from the MAC to PHY layer [25]. In the frame structure, up to four addresses are required to identify the WLAN access point address. These four fields enable to the registration of the access point addresses in the case of two users sending a packet in WLAN, each with a different access point [26].

In WLAN, all clients are using the same channel for transmission. According to this, the WLAN network standard requires a mechanism that determines how clients can or cannot send to the network. Multiple access mechanism enables to handle this issue. Such a mechanism is known as multiaccess with carrier avoidance (CSMA/CA). CSMA/CA enables client to work together to differ access to the medium using the same wireless channels [27].

### 3.1. QoS-Based Intelligent DCF Structure

Carrier-sense multiple access collision avoidances are based on the multiple access technique used in Ethernet connections that depends on collision detection [28]. In the CSMA mechanism, senders sense the first transmission channel and ensure that is not occupied by any other transmission. This mechanism helps avoid packet collisions with other senders. The mechanism of CSMA collision detection is used in wired Ethernet connections. It enabled to detection of collision occurrence. In wireless communications, the mechanism of collision detection is not possible [29]. The IEEE802.11 releases a standard to enable collision avoidance with a strategy of waiting and sending through shared wireless channels. IoT WLAN clients must ensure that the wireless channels have not been occupied for some time before they transmit their packets.  Figure 2 shows the proposed method QoS-based intelligent DCF that propose a waiting and sending mechanism according to the dynamic RT services [30–34].

### 3.2. QoS-Based PCF Structure

Point coordination function (PCF) is another protocol used as a part of IEEE 802.11 [35]. PCF enables two sensitive packets to allow for the transmission of data with higher priority over high data. The strategy of PCF depends on using the polling procedure that helps manage the free period for the priority over the DCF procedure. In the free period of PCF contention, a single host allows the clients to transmit their sensitive packets [36].

### 3.3. Enhanced Distribution Coordination Function (EDCF) for QoS

This paper proposed a new intelligent enhanced distribution coordination function based new QoS structure for the point coordination function that suites for dynamic real-time applications and services. The EDCF mechanism is provided to supply prioritized QoS by improving the contention-based DCF. EDCF gives separated, conveyed accessing remote media for QoS systems and devices and utilizes diverse user priorities [37]. The EDCF component characterizes four distinctive first-come, first-served (FCFS) lines (see Figure 3), called accesses categories (AC) [38] that give a bolster for the conveyance of activity with user priorities to the QoS systems and devices. Any information bundle from a higher layer at the side of a particular client's need esteem ought to be mapped into comparing AC concurring to Table 1 [39–43]. For the accesses categories, an enhanced variant of the DCF called an enhanced distribution channel accesses function (EDCA) contends for a transmission opportunity (TXOP) [44].

From Figure 3, each AC carries on a virtual node, which it competes for accessing the mediums and then begins its backoff procedure.After detecting the mediums, the virtual node still needs to wait at least for the shortest AIFS period. In EDCF, a modern sort of uncertainty is presented, the arbitraries IFSs (AIFSs), the input of DIFSs in DCFs [45]. All AIFSs are uncertainties interim with subjective duration as follows:

(1) $$\begin{array}{c} \text{AIFSs}\left[\text{AC}\right]=T_{s}x\text{AIFSNs}\left[\text{AC}\right]+\text{SIFS}, \end{array}$$

where AIFSNs[AC] is noted as the arbitrated IFSs and specified by the ACs and the physical structure and the *T*_s_ time slot is the length of a slot time (see Figure 4).

The ACS with the lowest AIFSs has the top priority. The values of AIFSs [ACs], CW_max_ [AC], and CW_min_ [AC], which are denoted as the QoS-based EDCF coefficients, are broadcast by the AP via a beacon frame [46]. The objective of utilizing various contention coefficients for various queues is to assign a low priority category with a lengthier time delay than a high precedence category, so the high precedence category is probably the medium to be accessed prior to the low priority category. An inner collision occurs when more than one ACs finish the back-off time simultaneously. In such a circumstance, a simulated collision handler in each QSTA permits the highest-priority ACs to send their frame, and the others execute a back-off procedure with an enlarged CWs value [47].

## 4. Dynamic WLANs Applications Methodology

Generating a simulation methodology that is corresponding to typical scenarios is one of the severe topics in network simulations. In such scenarios and simulations, the topology of the wireless network contained many network clients and APs (i.e., 20 nodes), an access point station, and a wireless server in the WLAN. The access point is associated with other systems and devices (see Figure 5); it assists as a destination for the flow traffic that is sent from the servers or sources [48]. All APs and clients are distributed in such a way that every node is capable of detecting and sensing the transmitters from any part of the collision domain of the WLAN. The mobility is selected randomly and is defined as the mobility from the trajectory option, which in this thesis, we design the mobility to be inside the range of simulation (the mobility can be seen in the white lines in Figure 5). The scenario in Figure 5 is suited for smart city-based internet-of-thing (IoT) services, that is, city control and monitoring rooms for environmental and security, unmanned transportations and vehicles, RT surveillances, and smart management system for energy.

## 5. Simulation Methodology and Parameters

The simulation environments are created by the OPNET® modeler and simulation environment (version 18.9.0) on the Windows® platform (Windows® 10). For the simulation, there are a few parameters that were configured, that is, the data rate was chosen 11 Mbps for IEEE 802.11e with 54 Mbps data rate for IEEE 802.11g. Several PHY and MAC parameter values used in our experiments are conferred to IEEE802.11e the typical parameters shown in Table 2 for IEEE802.11b and Table 3 for IEEE802.11g. The MAC and physical parameter values used in IEEE802.11e and IEEE802.11 g are the same except for IEEE 802.11g used extended rate PHY (802.11g) and data rate 54 Mbps. We have developed the simulation and run it for two hours in a dual quad-core processor with 1 GB memory for all scenarios and then benchmarked the achieved results.

For comparison of the performance between EDCF and DCF, two models were developed; medium access in the first model was maintained by EDCF as default, and in the second one, DCF procedure is performed at the data link layer (DLL) as shown in Table 4. Network simulation environment parameters were configured as a benchmark configuration that has been done for both other models. Complete conditions were stated in Tables 2 and 3 show the PHY and MAC parameters configurations utilized in simulation. The network evaluation for performance is modeled by evaluating both models one by one in the OPNET® simulation tool, and then the achieved results are compared.

In the EDCF case, the four traffics scenarios and classes have been applied to the data link layer from upper layers, which are conforming to ACs-0, ACs-1, ACs-2, and ACs-3, respectively [48] to assist the efficiency of the new proposed algorithm, which provide differential services that are mandatory for real-time (RT) applications. In the case of DCFs, it is not mandatory to offer differential services, which leads to no access class provisioning being needed. As a result, various applications have been configured using the profile applications for the model (i.e., EDCF procedure) for various access classes. In the first application, we named data, while inside, there were applications referred to database, e-mail, FTTP, and HTTP; in the next application, we used the voice application; and in the last application, we used video conference in high resolution. Details are shown in Table 4.

With the configuration application profile, client profiles were modeled and configured by using the three applications/scenarios. In the development of scenarios, 20 nodes were configured to utilize the network administration services chaotically. During the simulation running, we observed that all traffic data have the growth to plot the whole network activities in terms of the random number of packets exchanged per time unit. In EDCF, we change the point coordination function (PCF) and hybrid coordination function (HCF) by default to enable them after inserting the value of access category in all applications as shown in Table 5.

## 6. Evaluation Results and Discussion

The results have been generated using OPNET® simulation: first, we had identified IoT scenario for smart cities in Figure 5, and then the parameters have been identified as well. In phase 3, the proposed intelligent MAC protocol has been applied and implemented in the OPNET®. In phase 4, QoS data have been collected by simulating for some real-time traffics. In phase 5, results have been illustrated using MATLAB 2020®. The purpose of this part is to review and analyze the test and simulation results conducted. A detailed analysis is given here to benchmark the WLAN, EDCF, and DCF behaviors and performance in mobility for different scenarios based on WLAN approaches. The result presents in throughput, media access delay, data drop, and retransmission attempt for data, voice, and video, where the data refer to e-mail, FTTP, and HTTP.

### 6.1. Performance Analyses for IoT-Based IEEE 802.11e

From the simulation results, in Figure 6, it is shown that the data rate for DCF and EDCF in mobility because of general EDCF does not add priority to data. For data retransmission attempt, it is shown in Figure 7 DCF is better than EDCF for data retransmission in mobility scenario.In the first three minutes, the data retransmission attempt was shorter than others that because the back-off number was smaller (i.e., data drop) in the nodes. One can notice that there are slight variations between EDCF and DCF procedures in terms of retransmission attempts.

This little contrast suggests in general that the retransmission endeavors made in DCF conventions could be a bit lesser than EDCF protocol in portability.  Figure 8 shows that for the initial simulation momentthe MAC layer delay for DCF and EDCF functions increases equally, and then afterward,DCF grieves to be less delay than EDCF. . The increment within the intelligent IoT WLAN MAC layer accesses delay for each protocol is because of the increment within the hop number contending to get accesses of media. As shown in Figure 9, the data drop is increased gradually because of the high data transmitted. However, there is no big difference between them; it is better in the end EDCF.

For the voice scenario, as observed from Figure 10, the throughput of EDCF is higher than DCF, and this is due to the contention window of the voicein EDCF protocol is longer than in DCF; the throughput of voice in EDCF protocol reaches 24 kbps. The result showed a higher retransmission attempts of EDCF than DCF because of the high throughput of voice in EDCF and data drop as we will see in Figure 11, in the first three minutes, there were no the retransmission attempts, but after that, it isincreased dramatically in EDCF, the EDCF protocol retransmission attempts reach approximate 1.2 packets per second.

Moreover, Figure 12 shows that the delay metric in intelligent IoT WLAN MAC layer access for DCF is higher than EDCF. The high delay in DCF media accessdue tohigh number of nodes thta do not have priority to use long contention window (unlike EDCF with long CW).The EDCF protocol delay reachedupto 10 packets per second. For voice data drop, Figure 13 shows that the high data drop in the voice of EDCF is more than DCF, not only because the high throughput of voice in EDCF is greater than DCF but also because the differential services that can offer the priority-based method to handle several data types, but it is clear that the retransmission attempts is also high in voice in EDCF. The data drop using the EDCF protocol in voice reach approximately 62 kbps.

For the video scenario, Figure 14 shows that the throughput of the DCF is lesser than EDCF because the EDCF adds the contention window that gets big priority to video, which makes the throughput high than DCF. The throughput of EDCF can reach approximately 0.5 Mbps. The observation from Figure 15 is that the retransmission attempt in the video is high for EDCF with the difference of more than 0.05 packets in retransmission attempt because the big data dropped for EDCF. The retransmission attempts for EDCF in the video reach approximately 0.51 packets per second.

Moreover, one can notice that Figure 16 shows the intelligent IoT WLAN MAC layer delay for both DCF and EDCF, where the EDCF is less than DCF, because of the priority of EDCF; this means EDCF is better than DCF in media access delay. The EDCF protocol can reach approximately 0.42 packets per second.  Figure 17 shows that after simulation time of 120 secs, the drop data in EDCF increases rapidly, due to the differential service behavior of EDCF, which provides the priority-based method to handle several data types. DCF is lower dropped data when it compares to EDCF. The data drops for the EDCF protocol in video approximately reached 45 kbps.

### 6.2. Performance Analyses for IEEE 802.11g

In such a case, we compare the real-time application of IEEE 802.11 g-stander for 54 Mbps data rate for DCF and EDCF to find the best protocol for quality of service in WLAN in mobility. In the results discussed, the efficiency, data rate, retransmission attempt, medium accesses delays, and dropped of data for voice and video conference only, while we left the pure data as one can see that, no change have been observed for data in EDCF. It observes from Figure 18 that the data rate and capacity of EDCF and DCF are starting as a high capacity for three minutes EDCF degradation; EDCF reaches 100 kbps.

As shown in Figure 19, the high retransmission for EDCF than DCF because the high data dropped for EDCF as we will see in data dropped for voice; the retransmission attempts for EDCF protocol reach approximately 2.2 packets per second.  Figure 20 shows that media access delay for voice for the EDCF which is found the delay less than DCF, this means EDCF is better than DCF in medium accessed delay for RT voice.The medium accesses delays for EDCF protocol in voice went upto 0.38 packets per second.It can be observed from Figure 21 that the data dropped for EDCF is higher than DCF in the voice because of the service differentiation, which provides the priority; the data drop for voice reach approximately 110 kbps, the reason forthat the EDCF shows less performance compared to DCF in mobility for IEEE 802.11 g.This degradation in EDCF performance is due to the degradedof the throughput.

It has been noticed from Figure 22 that for the first two minutes, there is the same throughput for DCF and EDCF; after that, the EDCF has comparatively increased throughput than DCF because of the high priority for video. Therefore, the results are better with EDCF; the EDCF protocol for video reaches approximately 1.8 Mbps. From Figure 23 that retransmission attempt packets per second for DCF is fairly more than EDCF, the video retransmission attempts for EDCF protocol approximately reach 0.73 packets per second. Intelligent IoT WLAN MAC accesses delays from Figure 24, the initial of simulation, the MAC access have delays for the two functions i.e., DCF and EDCF, where the increasessimilarly for both, and after awhile, DCFs packets suffer from delays to be more than EDCF.

The increment within the medium-get-to-delay (MGD) for the two models and scenarios is because of the extended and increment of the number of nodes hop in the network competing to access the medium; the media access delay for video in EDCF protocol reaches approximately 0.11 packet per seconds. In Figure 25, the data dropped for DCF and EDCF; the data drop for DCF is increasing more than EDCF because the differential services that implement the priority feature and algorithm to handle several numbers of data types and high throughput/capacity/data rate for EDCF; the video data drop for the EDCF protocol reach approximately 17 kbps.

As overall performance output, the results from thecollected data were aimed to find the best protocol for IEEE 8021.11b and *g* thatguaranteed QoSin mobility scenario. We noticedthat the throughput metrics for real-time application in EDCF was better thanDCF in IEEE 8021.11b standard. That means, the EDCF is appropriate forreal-time applications i.e., voice and video conference.IEEE8021.11g showed that there different performancesfor voice and video throughputs; however in overall the EDCF was the more appropriatedthan DCF for real-time application in QoS in mobility.

## 7. Conclusions

Wireless local area networks recently get much interest among industry and academia researchers where many standards are coming out very fast. This fast grows results from a raised of the weaknessesofWLAN real-time applications quality that leads the nodes locked to deadlock or starvations. The future directions and challenges for 6G-enabled wireless communication for IoT applications are mainly focusing on the quality of services (QoS). The allocating of channel radios in WLAN for the higher needs activities is much more effective than for lower needs. Higher requirement activities made lower need activities that can be tolerated acceptable QoS. In terms of by and large execution (i.e., beneath the utilized recreation circumstances in the specific deliberate of QoS for WLAN), EDCF performs possibly less than DCF. This occurs because in EDCF nodes, all ACs perform like virtual systems and devices for media, so more packet collisions may be anticipated for EDCF situations.

The paper proposed a new QoS structure for the PCF that is based on an intelligent enhanced DCF that suites with dynamic RT IoT applications and services for the smart city, that is, RT surveillances, unmanned transportations and vehicles, smart management system for energy, city control, and monitoring rooms for environmental and security. In terms of quality of service (QoS) for real-time applications (i.e., video streaming or teleconferences), EDCF outperforms DCF. EDCFs frames have been aimed at the intelligent medium access control (IMAC) convention for IEEE standards growth and QoS standard IEEE802.11e. The remote gadgets utilizing EDCF as intelligent IoT WLAN MAC convention would be accessible in the showcase within another coming two long times. By and by, all remote devices, DCF is utilized as the default medium access protocol, and PCFS frames are utilized as the discretionary usefulness. For future work, it is recommended to check the performance with different values of nodes and access points, for example, thirty, fourth, fifty,… and so on. Additionally,it is recommended to applythe proposed technique to a different technologies, i.e., ad hoc, wireless sensor network. This paper has evaluated and tested through a large scale of the network of wireless nodes, and the throughput has been calculated utilizing OPNET® event-driven tool for network evaluation. The paper was modeled with limitations from different parameters and conditions such as the simulation tools limitation, simulation time, and limitations based on the microsystems memory and microprocessor used for running the OPNET®. The proposed ECDF algorithm can still be enhanced with less delay, packet drop, and throughput.

## Figures and Tables

**Figure 1:** Frame structure for packet access in MAC Layer.

**Figure 2:** The proposed QoS-based intelligent DCF for RT IoT applications.

**Figure 3:** Four AC transmission queue implementation models.

**Figure 4:** The timing relationship of EDCF.

**Figure 5:** The IoT WLAN network model with intelligent mobility scenario.

**Figure 6:** Data throughput in mobility.

**Figure 7:** Data retransmission attempts in mobility.

**Figure 8:** Data media access delay in mobility.

**Figure 9:** Data dropped.

**Figure 10:** Throughput for voice.

**Figure 11:** Retransmission attempt for voice in mobility.

**Figure 12:** Media access delay for voice in mobility.

**Figure 13:** The data dropped in voice in mobility.

**Figure 14:** The throughput for video in mobility.

**Figure 15:** Retransmission attempt in the video.

**Figure 16:** Media access delay in the video in mobility.

**Figure 17:** The data dropped in the video.

**Figure 18:** The throughput of voice.

**Figure 19:** Retransmission attempt for voice.

**Figure 20:** Media access delay for voice.

**Figure 21:** Data drop for voice.

**Figure 22:** Throughput for voice.

**Figure 23:** Retransmission attempts for video.

**Figure 24:** Video media access delay.

**Figure 25:** Data drop for real-time application, that is, video streamings.

**Table 1:** AC and TXOP access class details.

TXOP	AC	Description
1	0	Backgrounds
2	0	Standards
0	1	Best efforts
3	1	Exceptional efforts
4	2	Multimedia streaming (MMS)
5	2	Multimedia interactives (MMI)
6	3	Voice interactives (VI)
7	3	Unused

**Table 2:** PHY and intelligent IoT WLAN MAC coefficients that utilized in the simulation configurations for all scenarios.

Attribute	Values
Physical features	DS
Data rates	11 Mbps
Transmit powers	5 MW
Buffer sizes	256,000 bits
BSSs identifiers	Autoassign
Channels configurations	Autoassign
Roaming capabilities	Enabled
AP beacon interval (sec)	2 MW
Processing of large packets	Drops

**Table 3:** PHY and MAC parameters configurations utilized in the simulation for IEEE802.11 g.

Attribute	Value
Characteristics of the PHY layer	Extended rate PHY (802.11g)
Data rates	54 Mbps
Transmit powers	100 MW
Buffer sizes	256,000
BSSs identifiers	Autoassign
Channels configuration	Autoassign
Roaming capabilities	Enabled
AP beacons intervals	5 ms
Processing of large packets	Drops

**Table 4:** Access class matching to the applications.

Access classes	Applications configuration	Description
AC (0)	HTTPS (light-weight)	Backgrounds
AC (1)	Login remotely (heavy-weight)	Excellent efforts (EE)
AC (2)	Video conferencing	Interactive multimedia (IMM)
AC (3)	Voice over IP	Interactive voices (IV)

**Table 5:** The parameters for the access category.

Priority	AC	CW_min_	CW_max_	AIFSN
0	Voice	7	15	2
1	Video	15	31	2
2	Best effort	31	1,023	3
3	Background	31	1,023	7

## Data Availability

The data sets or codes generated during and/or analyzed during the current study are available from the corresponding author on reasonable request.
